The article "Mitochondrial-Endoplasmic Reticulum Communication-Mediated Oxidative Stress and Autophagy" was published in 2022. Journal: Biomed Res Int.

# Mitochondrial-Endoplasmic Reticulum Communication-Mediated Oxidative Stress and Autophagy

**DOI:** 10.1155/2022/6459585

**Published:** 2022-09-17

**Authors:** Xiaoqing Liu, Riaz Hussain, Khalid Mehmood, Zhaoxin Tang, Hui Zhang, Ying Li

**Affiliations:** ^1^College of Veterinary Medicine, South China Agricultural University, Guangzhou 510642, China; ^2^Faculty of Veterinary and Animal Sciences, The Islamia University of Bahawalpur, 63100, Pakistan

## Abstract

Oxidative stress is an imbalance between free radicals and the antioxidant system causing overgeneration of free radicals (oxygen-containing molecules) ultimately leading to oxidative damage in terms of lipid peroxidation, protein denaturation, and DNA mutation. Oxidative stress can activate autophagy to alleviate oxidative damage and maintain normal physiological activities of cells by degrading damaged organelles or local cytoplasm. When oxidative stress is not eliminated by autophagy, it activates the apoptosis cascade. This review provides a brief summary of mitochondrial-endoplasmic reticulum communication-mediated oxidative stress and autophagy. Mitochondria and endoplasmic reticulum being important organelles in cells are directly or indirectly connected to each other through mitochondria-associated endoplasmic reticulum membranes and jointly regulate oxidative stress and autophagy. The reactive oxygen species (ROS) produced by the mitochondrial respiratory chain are the main inducers of oxidative stress. Damaged mitochondria can be effectively cleared by the process of mitophagy mediated by PINK1/parkin pathway, Nix/BNIP3 pathways, and FUNDC1 pathway, avoiding excessive ROS production. However, the mechanism of mitochondrial-endoplasmic reticulum communication in the regulation of oxidative stress and autophagy is rarely known. For this reason, this review explores the mutual connection of mitochondria and endoplasmic reticulum in mediating oxidative stress and autophagy through ROS and Ca^2+^ and aims to provide part of the theoretical basis for alleviating oxidative stress through autophagy mediated by mitochondrial-endoplasmic reticulum communication.

## 1. Introduction

Oxidative stress is the imbalance between oxidative system and antioxidant system induced by internal and external environmental stress factors. It is generally believed that oxidative stress is mainly caused by strong oxidizing free radicals such as reactive oxygen and reactive nitrogen species, and the mitochondria respiratory chain is the main source and target of ROS. At the same time, mitochondrial oxidative stress also affects the transmission of redox signals through the mitochondrial-associated endoplasmic reticulum membrane. Finally, mitochondria and endoplasmic reticulum activate the autophagic pathways to alleviate oxidative damage. Autophagy is a process in which cells degrade proteins and damaged organelles through lysosomes, thereby promoting cell metabolism and maintaining a stable internal environment. Autophagy is an important pathway for cell regeneration and provides raw materials for synthesis of intracellular chemicals. At present, studies have found that autophagy inhibition will aggregate toxic proteins, cause cell apoptosis, and further lead to the occurrence of diseases [1]. PINK1/parkin is the main pathway that mediates mitochondrial autophagy, and mutations of PINK1 and parkin cause abnormal morphological and functional mitochondrial accumulation causing substantia nigra neurodegeneration and early-onset Parkinson's disease [2]. In addition, it has also been reported that excessive activation of mammalian target of rapamycin (mTOR) plays an important role in autophagy, regulates cell proliferation and metabolism, and promotes tumor development in terms of growth factor receptor signaling, lipid metabolism, cancer cell migration, and autophagy inhibition [3]. Moreover, Matsui et al. reported that autophagy is important for the regulation of heart homeostasis under stress conditions. The overexpression of AMPK and the forced activation of mTOR caused autophagy inhibition, which significantly aggravated the ischemic damage of the heart [4].

The article "Mitochondrial-Endoplasmic Reticulum Communication-Mediated Oxidative Stress and Autophagy" was published in 2022. Journal: Biomed Res Int.

ROS are the key and important factors among different oxidative stress inducing factors in the cells and are also closely related to autophagy. ROS can be used as signal molecules for autophagy. It is recorded that, during modification of Atg4, LC3BI can be converted into LC3BII and promotes the extension of autophagosome membranes [5]. In addition, reactive oxygen species increase autophagosome formation by inducing adenosine monophosphate-activated protein kinase (AMPK) phosphorylation, inhibiting mTOR, and activating uncoordinated 51-like kinase 1(ULK1) [6]. Studies have shown that exogenous hydrogen peroxide can increase the expression of Beclin1 and LC3 in Hela cells, thereby activating the process of autophagy [7], and increase levels of antioxidant enzymes can inhibit the occurrence of autophagy [8]. The regulation of autophagy also affects the level of oxidative stress in cells. Under the influence of some unfavorable factors, cells can promote dysregulated mitochondrial turnover through mitophagy and can also activate Nrf2 factor [9], regulate the activity of antioxidant enzymes, and maintain cellular redox homeostasis. Briefly, under oxidative stress conditions, reactive oxygen species can activate the process of autophagy, and autophagy alleviates oxidative damage to a certain extent by eliminating damaged organelles and degrading protein aggregates and reducing the production of reactive oxygen species.

The article "Mitochondrial-Endoplasmic Reticulum Communication-Mediated Oxidative Stress and Autophagy" was published in 2022. Journal: Biomed Res Int.

Communication between mitochondria and endoplasmic reticulum plays an important role in oxidative stress and autophagy. Their communication relies on a membrane structure formed between the endoplasmic reticulum membranes and the mitochondrial outer membranes. A variety of proteins with great significance in apoptosis, autophagy, lipid transport, mitochondrial dynamics, and Ca^2+^ signaling are located in mitochondria-associated ER membranes (MAMs). They not only structurally tightly connect mitochondria and endoplasmic reticulum but also undertake the material transport and signal molecule transmission between the two organelles [10]. This review for the first time explains the role of mitochondria, endoplasmic reticulum, and their communication in oxidative stress and autophagy. In addition, it also describes the link of ROS and Ca^2+^ as signaling molecules in mitochondria-endoplasmic reticulum communication in oxidative stress and autophagy.

## 2. Oxidative Stress

Oxidative stress is defined as the impact of the imbalance between ROS production and antioxidant biomarkers. With the in-depth development of research, oxidative stress is considered to be the imbalance between the oxidative system and the antioxidant system, and ROS is the main cause of oxidative stress. Mitochondria-endoplasmic reticulum communication-mediated oxidative stress is shown in Figure 1. At present, the well-researched sources of ROS are mitochondrial oxidative phosphorylation, NADPH oxidase, and adrenaline autooxidation [11]. The outer layer of ROS has one or more unpaired single electrons, resulting in its highly reactive ability to oxidize almost any large molecule in cells [12]. ROS target DNA in cells and cause modification in bases and single-strand or double-strand breaks of DNA molecules. The unpaired single electron in ROS is easy to bind to nucleophilic DNA molecules, which leads to the appearance of purine and pyrimidine derivatives resulting in wrong base pairing and coding in DNA replication, and the occurrence of gene mutation [13]. The oxidative damage induced by ROS in cells is also shown by the effects on protein molecules. Thiol group is the key group of proteins, which determines the structure and functions of proteins [14]. ROS can oxidize sulfhydryl groups and cause oxidative denaturation of proteins. Moreover, ROS attacks the amino groups in protein molecules to generate ammonia gas and carbonyl derivatives, accelerating the degree of protein oxidation. In addition, ROS can oxidize membrane lipids, destroy cell membranes, and lead to increased membrane permeability and harmful intermediate products such as malondialdehyde (MDA), which further damage cells [15]. ROS can also be used as signal molecules to trigger the apoptosis cascade. ROS can mediate cell apoptosis through death receptors. Death receptors are transmembrane protein receptors that are members of the tumor necrosis factor receptor (TNFR) superfamily. They can bind to related ligands and undergo structural changes, exposing the death domains that can bind to adaptor proteins, accumulating and activating the articulation proteins [16], which stimulates caspases and mediates apoptosis. The tumor necrosis factor receptor superfamily is all type I transmembrane glycoproteins. In addition to inducing cell apoptosis, there are some members that can cause cell proliferation and activation. The ligands of members of the tumor necrosis factor receptor superfamily are all transmembrane glycoprotein receptors, and these ligands constitute the tumor necrosis factor superfamily (TNF). The most known death ligand is FasL. FasL binds to the receptor Fas and undergoes trimerization. Its death domain binds to the death domain of the adaptor protein to activate caspase-8 and form a protein complex that can activate caspase-3 and mediate apoptosis through the caspase-3 cascade reaction [17]. Reactive oxygen species can also mediate apoptosis through the mitogen-activated protein kinase (MAPK) pathways. MAPK is an important apoptotic signal regulation pathway, and extracellular stimulation can promote or inhibit the process of apoptosis by activating the MAPK cascade reaction pathway. MAPK has four main subfamilies: extracellular signal-regulated kinase (ERK), p38 mitogen-activated protein kinase (p38MAPK), c-Jun amino-terminal kinase (JNK), and extracellular signal-regulated kinase 5 (ERK5). The signal transduction pathways involved in these types of molecules which regulate different functions. Extracellular signal-regulated kinases generally play an important role in cell growth and differentiation [18], while the redox-sensitive JNK and p38MAPK signal pathways are closely related to stress responses such as inflammation and apoptosis [19]. Stimulated by stress signals, JNK and p38MAPK can phosphorylate transcription factors such as P53, increase their transcriptional activity, lead to the expression of target genes, and induce apoptosis through proapoptotic proteins [20].

The article "Mitochondrial-Endoplasmic Reticulum Communication-Mediated Oxidative Stress and Autophagy" was published in 2022. Journal: Biomed Res Int.

In order to alleviate cell oxidative damage, ROS activate the Nrf2/Keap1 pathway to upregulate the expression of genes encoding antioxidant enzymes and reduce ROS levels through negative feedback regulation mechanisms [21]. Under normal circumstances, Keap1 forms a complex with Nrf2, and at the same time, Keap1 can bind to ubiquitin ligase to make Nrf2 ubiquitinated and lose its activity. When oxidative stress occurs, Keap1 is oxidized by ROS, and ubiquitin ligase cannot target ubiquitinated Nrf2. Activated Nrf2 transfers to the nucleus and upregulates genes encoding antioxidant enzymes [22]. The cellular antioxidant system consists of three parts. The first part includes enzymes that can independently catalyze the decomposition reactions, such as superoxide dismutase and catalase. Superoxide dismutase (SOD) plays an important role in the antioxidant process of cells. It can catalyze the disproportionation reaction and decompose superoxide which is harmful to cells into hydrogen peroxide and oxygen [23]. It has functions of antioxidation, antiaging, and protecting cells from damage [24]. Superoxide dismutase is an erythrocuprein, discovered in 1969. There are four family members of SOD including Cu/Zn-SOD, Mn-SOD, Fe-SOD, and Ni-SOD [25]. The four enzymes are distinguished according to the different metal prosthetic groups. Catalase (CAT) is a class of enzymes that can accelerate the decomposition of hydrogen peroxide into water and oxygen, thereby protecting cells from the attack of reactive oxygen species, which have the functions of alleviating inflammation, protecting antioxidant system, and strengthening the body's immunity [26]. Catalase uses iron porphyrin as its auxiliary group. It not only indicates the oxidation level of cells but also is used as an indicator for the identification of bacterial biochemical characteristics [27]. Generally, catalase is divided into three categories according to the difference of structure like monofunctional catalase, manganese catalase, and hydrogen peroxide-catalase. The second part is the substance regenerated by thioredoxin and thioredoxin after interacting with ROS, also known as the thioredoxin antioxidant system. This system has thioredoxin reductase (Trx-R), reduced coenzyme II (NADPH), and thioredoxin (Trx). Thioredoxin acts as a redox carrier through disulfide bonds and thiols in a variety of reactions and is an important enzyme activity regulator protein [28]. The redox of disulfide bonds can efficiently transfer electrons and is the main regulation mechanisms in the signal. Thioredoxin can interact with other antioxidant systems in the cells. Thioredoxin can activate 2-cysteine peroxidase and eliminate reactive oxygen species in the cell [29]. The function of thioredoxin reductase is to convert oxidized thioredoxin into a reduced form, so that it can continue to play the role of antioxidation, growth-promoting, antiapoptosis, and regulating the activity of transcription factors [30]. The third part is composed of glutathione peroxidase 1, glutathione peroxidase 4, and glutathione. Generally, the ratio of reduced and oxidized glutathione is used to evaluate the degree of redox [31]. They use different ways to convert harmful ROS in the mitochondria into water and oxygen and ultimately reduce the oxidative damage of the mitochondria [32]. They use different ways to convert harmful ROS in the mitochondria into water and oxygen, and ultimately reduce the oxidative damage of the mitochondria [33]. Glutamate, cysteine, and glycine are precursors for the synthesis of glutathione. The synthesis process requires the regulation of glutamate-cysteine ligase and glutathione synthase. The basic form of glutathione peroxidase oxide can be eliminated by reduced glutathione. The hydrogen peroxide that is broken down by glutathione needs the catalysis of glutathione peroxidase (GPx).

The article "Mitochondrial-Endoplasmic Reticulum Communication-Mediated Oxidative Stress and Autophagy" was published in 2022. Journal: Biomed Res Int.

### 2.1. Mitochondrial Pathway-Mediated Oxidative Stress

Mitochondria is one of the most vital organelles in the cells. It is the main place for aerobic respiration. Mitochondria use tricarboxylic acid cycle and oxidative phosphorylation to convert sugar, fat, and proteins into energy, which helps the cells function normally. Besides, mitochondria can synthesize cholesterol and some heme, regulate cell proliferation and metabolism, regulate membrane potential, and control cell death. Mitochondrial regulation of cell death is closely related to the production of ROS during aerobic respiration. ROS is generally considered to be a pathogen produced by neutrophil to protect against injurious attack, but recent studies have found that ROS can also play a central role as a second messenger in determining the fate of cells and modifying various signaling molecules [34]. Mitochondria are the main source of ROS production, and high levels of ROS can also cause mitochondrial dysfunctions, leading to neurodegeneration and ischemic damage to the heart and brain [35].

ROS are mainly produced by electron transport in the respiratory chain of mitochondria. The electron transfer in mitochondrial respiratory chain is mainly carried out by the respiratory chain complex I (NADH-coenzyme Q reductase), II (succinate-coenzyme Q reductase), III (coenzyme q-cytochrome reductase), and IV (cytochrome c oxidase) and some free enzymes [36]. NAPDH and FADH_2_ in the tricarboxylic acid cycle supply electrons to the respiratory chain and are received by coenzyme Q and cytochrome C. When the electrons are transferred, a portion of the proton is pumped through the respiratory chain complex from the mitochondrial matrix to the outer membrane and the inner membrane, creating a potential difference between inside and outside the inner mitochondrial membrane. It is an important part of the respiratory chain, where the oxidative phosphorylation stores energy [37]. During normal respiration, about 90 percent of the oxygen is reduced to water via mitochondrial electron transport chain, and a small fraction of the escaped single electrons continue to be reduced to superoxide anion and hydrogen peroxide. The escaping single electrons mainly come from complex I and complex III [38]. In addition to oxidation, ROS can trigger the opening of mitochondrial permeability transition pore and release more ROS from mitochondria, causing different degrees of cell damage. This is a positive feedback mechanism, also known as ROS-induced ROS release (RIRR) [39].

The article "Mitochondrial-Endoplasmic Reticulum Communication-Mediated Oxidative Stress and Autophagy" was published in 2022. Journal: Biomed Res Int.

The type and quantity of proteins determine the diversity of mitochondrial functions, and the stability of proteins in mitochondria is the basis for maintaining mitochondrial morphology and function. The mitochondrial genome can encode more than 1,200 proteins, of which 13 are encoded in the mitochondria, and the remaining mitochondrial proteins are encoded in the nucleus, synthesized in the cytoplasm, and finally, directed to the mitochondria [40]. Under the influence of unfavorable factors such as hypoxia and oxidative stress, the signal transduction pathway in the mitochondria is damaged. A large number of unfolded and misfolded proteins accumulate in the mitochondria, causing toxicity, further aggravating the burden of mitochondria, and affecting the normal physiological functions of mitochondria. When damage to mitochondrial protein occurs, mitochondria induce mitochondrial molecular chaperones and proteases through signal transduction pathways to increase glycolysis and amino acid metabolism, inhibit tricarboxylic acid cycle and oxidative phosphate gene expression, and maintain protein stability state [41, 42].

### 2.2. ATF5-CHOP-Mediated Mitochondrial Unfolded Protein Response

Mitochondria receive the signal of protein toxic stress, activate CHOP transcription through the JNK pathway, and induce mitochondrial unfolded protein response. In the process of mitochondrial stress, transcription factor 5 (ATF5) transfers from mitochondria to the nucleus and interacts with DVE1 and VBL5 [43] and enhances the expression level of mitochondrial chaperone protein and protease. Mitochondrial chaperone proteins can promote the folding of unfolded proteins and prevent the accumulation of misfolded proteins. Protease can hydrolyze and remove damaged and misfolded proteins, preventing them from toxic to mitochondria [44]. The increased expression of chaperone proteins mainly consists of heat shock protein 60, heat shock protein 10, heat shock protein 70, and heat shock protein 90 [45]. Heat shock proteins 60 and heat shock protein 10 mainly mediate protein folding and assembly. Heat shock protein 70 and heat shock protein 90 help the transfer of mitochondrial protein precursors from the cytoplasm to the mitochondrial matrix.

The article "Mitochondrial-Endoplasmic Reticulum Communication-Mediated Oxidative Stress and Autophagy" was published in 2022. Journal: Biomed Res Int.

### 2.3. Sirt3-FOXO3a-Mediated Mitochondrial Unfolded Protein Response

Silent information regulator 3 (Sirt3) belongs to the family of nicotinamide adenine dinucleotide-dependent histone deacetylases. It participates in the regulation of cell metabolism, aging, and apoptosis by regulating important cellular physiological processes such as the tricarboxylic acid cycle and fatty acid oxidation [46]. FOXO3a belongs to the O subtype of the fork-head transcription factor. It can target mitochondria and nuclei to upregulate the expression of SOD1, SOD2, and CAT, reduce the content of reactive oxygen species, and play an antioxidant role. The content of reactive oxygen species in the mitochondria is reduced, and the degree of oxidative stress is reduced, which is conducive to reducing the number of unfolded and misfolded proteins and maintaining the normal function of mitochondria. Sirt3 plays a very important role in mitochondrial metabolism. ROS can promote the transcription of FOXO3a by activating Sirt3, thereby regulating the genes of SOD and CAT.

### 2.4. ER*α*-Mediated Mitochondrial Unfolded Protein Response

Unfolded and misfolded proteins in mitochondria promote the increase of reactive oxygen species in mitochondria, protein kinase Akt is phosphorylated [47], estrogen receptor (ER*α*) is activated, and nuclear respiration factor 1 (NRF1) and high temperature demand protein A2 (HTRA2) are promoted. The transcription further improves the expression of protease [48]. The above three pathways that mediate the unfolded protein response have a synergistic effect. When one of the pathways is inhibited, the signal molecules that mediate the other pathways will be activated and exert their compensatory effects.

### 2.5. Mitochondrial-Endoplasmic Reticulum Pathway-Mediated Oxidative Stress

Endoplasmic reticulum (ER) is an indispensable organelle in cells, which can synthesize and modify proteins, anabolic steroids and lipids. At the same time, endoplasmic reticulum is the largest calcium pool in cells. The endoplasmic reticulum membrane has many Ca^2+^ channels, in which the ryanodine receptor (RyR) and the 1,4,5-inositol triphosphate receptor (IP3R) are in the endoplasmic reticulum. Ca^2+^ main passages for outward transport-Ca^2+^ pumps (Ca^2+^- ATPase) and Ca^2+^-binding proteins are responsible for most of the recovery of endoplasmic reticulum from cytoplasm Ca^2+^ to get to the bottom of this. When the endoplasmic reticulum is stimulated, the receptor phosphatase C (PLC), an enzyme that cleaves the endoplasmic reticulum membrane phosphatidylinositol 4,5 diphosphate (P2), is activated. Inositol 1,4,5-triphosphate (IP3) is produced by enzymatic hydrolysis of P_2_ and can bind and activate IP3R [49]. Ca^2+^ from IP3R is released out of the endoplasmic reticulum and is regulated by GRP75, a protein molecule, from the voltage-dependent anion channel (VDAC) on the outer mitochondrial membranes and the mitochondrial calcium unidirectional transport protein on the mitochondrial matrix [50]. This channel significantly improves the efficiency of calcium ions entering the mitochondria. Ca^2+^ have been shown to increase the activity of some important enzymes in tricarboxylic acid cycle, enhance respiratory chain function, and promote ATP production [51]. In this case, the increase of ROS produced by mitochondria induced the opening of mitochondrial permeability transition pore. ROS are released into the mitochondria via the MPTP, causing oxidative stress in cells.

The article "Mitochondrial-Endoplasmic Reticulum Communication-Mediated Oxidative Stress and Autophagy" was published in 2022. Journal: Biomed Res Int.

In addition to direct oxidative damage, ROS acts as a second messenger to the endoplasmic reticulum to regulate calcium transport. On the one hand, ROS can damage RyR and IP3R gating, opening up channels that transport Ca^2+^ to mitochondria and cytoplasm [52]. On the other hand, ROS suppression Ca^2+^- ATPase activity, resulting in the endoplasmic reticulum recycling of free Ca^2+^ blocked. Therefore, ROS can cause the disorder of Ca^2+^ homeostasis in the endoplasmic reticulum, thus impeding the synthesis and release of proteins. A large number of unfolded and misfolded proteins accumulate in the endoplasmic reticulum cavity, increasing the load of the endoplasmic reticulum and causing endoplasmic reticulum stress. As Ca^2+^ is transported through the MCU to the mitochondrial matrix, the mitochondria become overloaded with Ca^2+^ and more ROS, creating a vicious cycle.

When excessive amount of toxic proteins accumulates in the endoplasmic reticulum, these trigger an unfolded protein response to deal with endoplasmic reticulum stress. The unfolded protein reaction usually starts with the activation of PERK (PKR-like ER kinase), IRE1 (inositol-requiring enzyme1), and ATF6 (activation transcription factor 6) [53]. PERK is a protein kinase located in the endoplasmic reticulum membrane that can receive stress signals. When the endoplasmic reticulum is in a nonstressed state, it is inactive because its dimerization sites are covered. When the endoplasmic reticulum is under stress, GRP78 dissociates from PERK, and PERK is activated, which makes eIF2*α* autophosphorylate the site that initiates protein translation, and reduces the level of protein translation, which reduces the burden on the endoplasmic reticulum [54]. In addition, PERK can also regulate the antioxidant response by activating Nrf2. IRE1 is an endonuclease with kinase and RNase activity, belonging to the endoplasmic reticulum type I transmembrane glycoproteins. IRE1 can accept the signals of misfolded protein accumulation and transmit this signal across the membrane. Under normal circumstances, IRE1 is inactive and interacts with GRP78 [55]. When endoplasmic reticulum stress occurs, IRE1 is phosphorylated to activate RNase activity. The mRNA of XBP1 is cut and reconnected before it can be effectively translated [56]. XBP1 is a transcription factor that can enter the nucleus and activate genes involved in reduced protein synthesis and degradation of the endoplasmic reticulum-related molecules, thereby reducing endoplasmic reticulum stress [57]. ATF6 is a type II transmembrane protein on the endoplasmic reticulum. When the unfolded protein of the endoplasmic reticulum accumulates, ATF6 separates from GRP78, is transferred to the Golgi apparatus, and produces free fragments in the nucleus to enhance the expression of molecular chaperone genes in the endoplasmic reticulum, increase protein folding, and reduce endoplasmic reticulum stress [58].

The article "Mitochondrial-Endoplasmic Reticulum Communication-Mediated Oxidative Stress and Autophagy" was published in 2022. Journal: Biomed Res Int.

## 3. Autophagy

Mitochondria-endoplasmic communication-mediated autophagy is shown in Figure 2. The generation of autophagosomes is divided into three steps: nucleation, extension, and closure. The ULK1 complex and PI3KC3 complex are the key factors to the nucleation of phagocytic vesicles. ULK1 complex is composed of ULK1, FIP200, Atg13, and Atg101 [59]. During starvation, mitochondrial dysfunction or, in the presence of pathogens, Atg13 is dephosphorylated, enhancing the interaction between ULK1 and Atg101. Atg101 is a stabilizer of Atg13 and ULK1, which can effectively prevent the degradation of Atg13 proteasome, enable the ULK1 complex to initiate the formation of phagocytic vesicles, and recruit autophagy-related proteins to complete the extension and closure of autophagosomes [60]. Another activator closely related to autophagy is the PI3KC3 complex. The PI3KC3 complex is composed of PI3KC3, PIK3R4, Atg14, and Beclin1. The ULK1 complex phosphorylates Beclin1 and recruits and phosphorylates Atg14 [61]. Atg14 improves the interaction between phosphorylated Beclin1, PI3KC3, and PIK3R4 and enhances the activity of PI3KC3 lipid kinase, which releases PI3P and recruits more autophagy-related proteins to form autophagosomes [62]. The PI3KC3 complex binds to Atg16, and the Atg16-Atg5-Atg12 complex binds phosphatidylethanolamine (PE) and LC3 to form LC3II and position the autophagy membrane at the position of LC3 [63]. Autophagosomes fuse with lysosomes to form autophagolysosomes. Therefore, LC3 is often used as a marker to detect the level of autophagy [64].

The article "Mitochondrial-Endoplasmic Reticulum Communication-Mediated Oxidative Stress and Autophagy" was published in 2022. Journal: Biomed Res Int.

Autophagy, as a way of process of cell self-renewal, has attracted much attention since it was discovered in 1950. Studies have found that the autophagy pathway not only has its own genes but also communicates with almost all signal networks and organelles in the cells, which is the key to the normal function of the cell [65]. When cells are oxidatively stimulated, they can induce autophagy through the AMPK-mTOR-Nrf2 pathway and regulate autophagy according to the level of oxidation [66]. As mentioned above, oxidative stress can phosphorylate Keap1, leading to the accumulation of Nrf2 and enhancing the expression of genes of antioxidant enzymes. In addition, oxidative stress can also phosphorylate P62, enhance its ability to bind to Keap1, and transfer Nrf2 to the nucleus to play a role [67]. Nrf2 can activate autophagy-related genes when the level of oxidation increases. The process of autophagy requires the regulation of autophagy-related genes (Atgs) and requires AMPK and mTOR to conduct signaling molecules. Under mild oxidative conditions, AMPK is activated and mediates autophagy by inhibiting mTOR [68]. However, under high levels of oxidative stimulation, the expression of Nrf2 is abnormally active, but the activity of AMPK is downregulated. However, some researchers have reported that under high levels of oxidative stress, Nrf2 inhibits AMPK activity and prevents AMPK overexpression from inducing apoptosis, and mTOR can inhibit Nrf2. This double-negative feedback ensures the stability of the autophagy regulatory mechanisms [69]. Although autophagy is the process of cell self-renewal and if autophagy cannot keep the cell steady, it will lead to apoptosis. For example, under normal circumstances, Bcl2 binds to Beclin1 and Bax to inhibit autophagy and apoptosis. During the starvation, JNK is activated and phosphorylates Bcl2, Beclin1 is released, and autophagy is induced [70]. When the body is in a state of long-term starvation, phosphorylated Bcl2 binds to Bax to inhibit cell apoptosis. But during the extreme starvation, JNK promotes the separation of Bcl2 from Bax, and then, Bax induces cell apoptosis through the caspase3 pathway [71].

### 3.1. Mitochondrial Pathway-Mediated Autophagy

When mitochondria are influenced under the action of different factors, cells can selectively degrade the damaged mitochondria through the mediation of receptors protein or adaptor protein, to avoid the overflow of apoptosis-inducing molecules in mitochondria, in order to maintain the normal activities of the cells [72]. Early studies on autophagy were carried out using yeast, and it was found that yeast can also undergo mitochondrial autophagy in the context of starvation and that mitochondrial targeting proteins were found in yeast [73]. One of the most important proteins is Atg32, which interacts with Atg8 to induce autophagosomes to migrate to damaged mitochondria, where they degrade to small molecules [74]. There are multiple pathways in mammalian cells that enable autophagosomes to recognize damaged mitochondria.

The article "Mitochondrial-Endoplasmic Reticulum Communication-Mediated Oxidative Stress and Autophagy" was published in 2022. Journal: Biomed Res Int.

### 3.2. PINK1/Parkin Pathway-Mediated Mitochondrial Autophagy

PINK1 is present in the cytoplasm and then transported to the inner mitochondrial membrane by a transporter, which is broken down and inactivated by presenilin-associated rhomboids in the endometrium. This results in a low level of PINK1 in mitochondria under normal conditions. When the mitochondria are damaged by oxidation, the mitochondrial membrane potential decreases. PINK1 cannot normally bind to the mitochondrial inner membrane, but it can still combine with the mitochondrial outer membrane, which results in a large amount of PINK1 [75]. It cannot be hydrolyzed and accumulates in the outer mitochondrial membrane. PINK1 phosphorylates ubiquitin ligase in the cytoplasm, and Parkin autocatalytic mechanism amplifies this activation [76]. Activated Parkin is recruited into mitochondria and promotes ubiquitination of various proteins on the mitochondrial membrane [77]. The ubiquitinated membrane protein bound to the receptor protein P62 and used as a marker to localize the damaged mitochondria and mediate the autophagy of the damaged mitochondria. Genetic experiments on fruit flies have shown that PINK1 and Parkin work together to regulate mitochondrial functions, and the loss of any one of these proteins can lead to mitochondrial dysfunction, resulting in the degeneration of muscles and neurons in drosophila while overexpression of Parkin can improve the symptoms of PINK1 deletion [78].

### 3.3. Nix/BNIP3 Pathway-Mediated Mitochondrial Autophagy

BNIP3 is widely expressed in almost all human cells and is a well-known member of the BNIP family. BNIP3 is less abundant in cells, but increases in hypoxia. Hypoxia-inducible factor-1(HIF1) is an important nuclear transcription factor in hypoxia-induced apoptosis, which can directly regulate the expression of BNIP3 [79]. High expression of BNIP3 can induce mitochondrial autophagy, and excessive mitochondrial autophagy can induce apoptosis. BNIP3 is involved in every process of mitochondrial autophagy. In the initial stage of mitochondrial autophagy, due to the influence of unfavorable factors, BNIP3 is activated, thereby inhibiting the regulatory effect of mTOR, thus mediating mitochondrial autophagy. BNIP3 has a strong affinity to autophagy-related protein LC3 and can bind to mitochondria in the form of dimer to activate autophagy [80]. The results showed that the phosphorylation of BNIP3 promotes the interaction between LC3b and GATE-16 and enhances mitochondrial isolation, autophagy transmission, and degradation [81]. In addition, the expression of BNIP3 also promoted the free release of Beclin1 protein. The specific mechanism is that BNIP3, a homologous domain BH3 with Bcl_2_, can compete with Beclin-1 for the binding site of Bcl_2_ and promote the separation of Beclin1 from Bcl_2_, by binding to mitochondria. Beclin1 forms a complex with type III PI3K, which regulates the localization of downstream autophagy-associated proteins in the autophagy precursors and activates the autophagy of mitochondria [82]. However, BNIP 3 may also directly induce apoptosis via Bcl_2_ pathway. Nix is the homologous protein of BNIP3. Nix overexpression can decrease the mitochondrial membrane potential and induce Parkin to migrate to mitochondria, thus activating PINK1/Parkin pathway-mediated mitochondrial autophagy [83].

The article "Mitochondrial-Endoplasmic Reticulum Communication-Mediated Oxidative Stress and Autophagy" was published in 2022. Journal: Biomed Res Int.

### 3.4. Mitochondrial Autophagy Mediated by FUNDC1 Pathway

FUN14 domain protein 1(FUNDC1), a recently discovered molecule that mediates mitochondrial autophagy, is a triple-helix transmembrane domain with a sequence that interacts with LC3, known as the LC3 interaction region (LIR). Reversible phosphorylation of LIR is important for the activation of mitochondrial autophagy pathway by Fundc1 [84]. During normal conditions of oxygen content, SER13 and Tyr18 of Fundc1 are highly phosphorylated, while under the stimulation of hypoxia and mitochondrial oxidative phosphorylation uncoupler (FCCP), FUNDC1 was dephosphorylated [85]. Compared with phosphorylated FUNDC1, dephosphorylated FUNDC1 has a better affinity to LC3 and promotes autophagic body localization to damaged mitochondria [86]. However, other studies have shown that during hypoxia, serine kinases ULK1 and ULK2 are recruited into damaged mitochondria and bind to the outer mitochondrial membrane receptor FUNDC1, phosphorylating Ser17, which enhances the interaction between FUNDC1 and LC3, to induce mitochondrial autophagy [87].

### 3.5. Endoplasmic Reticulum Pathway-Mediated Autophagy

Under stress conditions, the endoplasmic reticulum can induce unfolded protein response to clear up misfolded and unfolded proteins. When the endoplasmic reticulum cannot be maintained at steady state, the accumulated toxic proteins are degraded by proteasome and autophagy of the unfolded protein response to reduce endoplasmic reticulum stress-induced apoptosis.

The article "Mitochondrial-Endoplasmic Reticulum Communication-Mediated Oxidative Stress and Autophagy" was published in 2022. Journal: Biomed Res Int.

### 3.6. Endoplasmic Reticulum Autophagy Induced by UPR

Because oxidative stress to the endoplasmic reticulum was caused by different degrees of damage, the degree of cell response is also different. Endoplasmic reticulum stress can maintain the normal functions of the endoplasmic reticulum by activating the unfolded protein response to remove both unfolded and misfolded proteins. When the accumulation of deleterious proteins exceeds the endoplasmic reticulum clearance, apoptosis is induced by signaling molecules. Under normal conditions, the three proteins that trigger endoplasmic reticulum stress normally bind to the protein molecular partner, GRP78, and are inactive. When endoplasmic reticulum stress occurs, GRP78, PERK, eIF 2*α*, and ATF6 detach, helping unfolded proteins to form spatial structures [88]. The expression of autophagy-related genes such as ATG4, ATG5, and ATG12 was upregulated by the phosphorylation of eIF 2*α* by activated PERK [89]. In addition, the expression of CHOP induced by eIF 2*α* decreased the formation of Beclin1-Bcl2 complex, increased the free Beclin1, and enhanced endoplasmic reticulum autophagy. Another way in which CHOP induces autophagy is to increase the expression of LC3 by localizing more autophagosomes to the damaged endoplasmic reticulum (ER) and then degrading ER fragments. The unfolded protein activates IRE1 and forms a complex with ASK1-TRAF2 to activate JNK signaling pathway, which increases free Beclin1 and induces autophagy [90]. ATF6 is transferred to the Golgi region during stress; site1 and site2 proteins cleave ATF6 and upregulate the expression of death-related protein kinase 1 (DAPK1) [88]. DAPK1 can phosphorylate Beclin1, thereby mediating autophagy. The researchers found that cells that had been knocked out of the three key genes thought to mediate the endoplasmic reticulum-unfolded protein response were treated with either undilutin or carotene and found that ATF6 and PERK were absent; autophagy was similar to that of wild-type cells, but was significantly inhibited in IRE1-deficient cells [91]. This suggests that endoplasmic reticulum autophagy induced by unfolded proteins is more closely related to the expression of IRE1 gene.

### 3.7. Endoplasmic Reticulum Autophagy Induced by Calcium Pathway

In addition to endoplasmic reticulum autophagy, which can be induced by unfolded protein response, intracellular calcium concentration also plays a key role in endoplasmic reticulum autophagy. Ca^2+^ releases from the endoplasmic reticulum into the cytoplasm, activating kinases and proteases involved in autophagy. Carotene-induced endoplasmic reticulum stress, followed by activation of unfolded protein response, decreased protein synthesis, induced calcium-dependent autophagy, and increased LC3 expression and RNA inhibitors are then used to demonstrate that calcium-mediated autophagy is accomplished by activating AMPK, further inhibiting the expression of mTOR [92]. mTOR is a serine/threonine kinase and plays a key role in autophagy. Activated mTOR phosphorylates ULK 1 and ULK 2 and inhibits autophagy by blocking the interaction between ULK complex and AMPK. In addition, mTOR prevents autophagy by inhibiting the phosphorylation of Beclin1 by AMPK [93].

The article "Mitochondrial-Endoplasmic Reticulum Communication-Mediated Oxidative Stress and Autophagy" was published in 2022. Journal: Biomed Res Int.

### 3.8. Endoplasmic Reticulum Autophagy Induced by FAM134B

FAM134B is the first endoplasmic reticulum autophagy receptor found in mammals and is a homology of ATG40 in yeast cells [94]. FAM134B promotes fragmentation of the damaged endoplasmic reticulum by interacting with the LC3/GABARAP complex [95], produced endoplasmic reticulum stress, increased calcium concentration in cytoplasm, and calmodulin-activated CAMK2B. CAMK2B can promote the oligomerization of the phosphorylated FAM134B SER151, drive the endoplasmic reticulum to decompose into small fragments, and then, mediate autophagy through LC3 pathway [96].

## 4. Mitochondrial-Endoplasmic Reticulum Pathway-Mediated Autophagy

Mitochondria and endoplasmic reticulum are two important organelles in cells, which are closely linked in function and structure (Table 1). About 20% of the mitochondrial surface was found to be in contact with the endoplasmic reticulum membrane, known as the mitochondrial-associated endoplasmic reticulum (MAMs). Many proteins are related to the function of mitochondria and endoplasmic reticulum, such as MAMS, PINK1, and IP3R. Some regulatory signals between organelles are transmitted from this tight junction more efficiently than they are diffused through the cytoplasm [49]. Vesicular-associated membrane-associated protein (VAPB) is a recombinant protein on the endoplasmic reticulum membrane; it binds to the outer mitochondrial membrane protein tyrosine phosphatase protein 51(PTPIP51), forming a frenulum that connects the endoplasmic reticulum to the mitochondria and holds them at distances between 10 and 30 nm [97]. When VAPB or PTPIP51 is overexpressed, the contact surface between mitochondria and endoplasmic reticulum increased, resulting in calcium overload in mitochondria, opening of MPTP, release of cytochrome c and ROS, and induction of cell apoptosis. When the expression of VAPB and PTPIP51 was decreased, the distance between mitochondria and endoplasmic reticulum became longer, which led to the deficiency of Ca^2+^ in mitochondria, the inhibition of tricarboxylic acid cycle, and the decrease of ATP production. Moreover, Ca^2+^ in endoplasmic reticulum induce autophagy by activating AMPK and inhibiting the expression of mTOR [98]. In addition, there are many autophagy-related proteins in MAMs.

The article "Mitochondrial-Endoplasmic Reticulum Communication-Mediated Oxidative Stress and Autophagy" was published in 2022. Journal: Biomed Res Int.

## 5. Conclusion

The mitochondrial-associated endoplasmic reticulum membrane binds to the fats of the two organelles. Mitochondria are the most vulnerable organelles to oxidative stress, and because of the close relationship between mitochondria and endoplasmic reticulum, the dysfunctions of mitochondria lead to endoplasmic reticulum stress. In order to avoid oxidative stress leading to apoptosis, autophagy is activated by phagocytosis and degradation of damaged organelles [5]. In addition, MAMs play an important role in lipid metabolism, mitochondrial dynamics, inflammation, and antiviral activity. Changes in proteins in MAMs affect the development of some diseases. Therefore, MAMs can be used as an effective target for treatment therapy for different diseases such as cancer, neurodegeneration, and diabetes.

## Figures and Tables

**Figure 1:** Mitochondria-endoplasmic reticulum communication-mediated oxidative stress. When stimulated by starvation, hypoxia, etc., the ROS produced by the mitochondrial respiratory chain increases leading to oxidative stress. At the same time, ROS damages the Ca^2+^ channels in the endoplasmic reticulum and depletes the Ca^2+^ in the endoplasmic reticulum. The overload of Ca^2+^ in the mitochondria affects the production of ROS in the respiratory chain. In order to alleviate oxidative damage, mitochondria and endoplasmic reticulum can promote unfolded formation of spatial structure and misfolded proteolysis through unfolded protein reaction. (1) The accumulation of ROS and harmful proteins can activate JNK, thereby increasing the expression of CHOP and ATF5 transcription factors, encoding heat shock proteins and proteases that can hydrolyze misfolded proteins. (2) ROS increase the transcription of NRF1 by activating ER*α*, augment the expression of protease, and reduce oxidative damage. (3) Mitochondria can also enhance the levels of antioxidant enzymes SOD and CAT by activating the Sir3-FOXO3a pathway to protect cells from oxidative attacks. (4) Mitochondria can also improve the levels of antioxidant enzymes SOD and CAT by activating the Sir3-FOXO3a pathway to protect cells from oxidative attacks.

**Figure 2:** Mitochondria-endoplasmic communication-mediated autophagy. Mitochondria and endoplasmic reticulum can control the distance between the two organelles through PTPIP51 and VAPB protein, thereby affecting the Ca^2+^ exchange between mitochondria and endoplasmic reticulum. Ca^2+^ is the second messenger in cells, and its content can regulate the degree of oxidative stress and autophagy of mitochondria and endoplasmic reticulum. (1) When oxidative stress occurs, the mitochondrial membrane potential decreases, PINK/parkin pathway is activated, and membrane proteins are ubiquitinated. Ubiquitinated membrane proteins bind to LC3 and p62 to localize autophagosomes to damaged mitochondria. (2) Mitochondria can also activate ULK1 complex and PIK3C3 complex by phosphorylating Beclin1 and inhibiting mTOR to enhance the expression of autophagy genes and promote the formation of autophagosomes. (3) The FUNDC1 receptor on the mitochondrial membrane has a good affinity with ULK1 and can bind to it to induce mitochondrial autophagy. (4) The endoplasmic reticulum-unfolded protein response can phosphorylate eIF2*α* by activating PERK, thereby promoting the expression of autophagy-related genes and enhancing the transcription of CHOP, thereby recruiting autophagosomes. IRE1 can also increase the expression of CHOP transcription factors by activating JNK. ATF6 can upregulate the activity of death-related proteases, phosphorylate Beclin1, and induce autophagy. (5) Increased Ca^2+^ in the cytoplasm can activate CAMK2B, thereby activating AMPK and inhibiting the phosphorylation of mTOR. (6) The combination of FAM134B and LC3 accelerates the fragmentation of damaged endoplasmic reticulum and promotes the formation of autophagic membranes.

The article "Mitochondrial-Endoplasmic Reticulum Communication-Mediated Oxidative Stress and Autophagy" was published in 2022. Journal: Biomed Res Int.

**Table 1:** Mitochondria-endoplasmic reticulum-related regulatory proteins and associated functions.

Related proteins	Function	Literature
FUNDC1-IP3R complex	Enhances the connection between mitochondria and ER and promotes Ca^2+^ flow to mitochondria.	[99]
MFN2	Deletion of MFN2 enhances contacts between the ER and mitochondria, promoting mitochondrial uptake of Ca^2+^.	[100]
TOM40-TOM70	Directing Atg2A to MAMs to mediate expansion of phagocytic vesicles.	[101]
IP3R-GRP75-VDAC1	GRP75 binds to IP3R and VADC, enhances the stability of the complex, and improves the efficiency of Ca^2+^ transport.	[102]
Sig-1R	Regulation of autophagosome-lysosome fusion.	[103]
BAP31	Inhibition of BAP31 expression can activate the AMPK-ULK1-LC3 pathway to induce autophagy.	[104]
FATE1	Promotes Ca^2+^ transfer from ER to mitochondria.	[105]
AMBRA1	AMBRA1 binds to the Beclin1 complex and promotes the autophagy cascade. In addition, it can also bind to lipid rafts such as GD3 and WIPI1 and positively regulate autophagy.	[102]
PACS-2	Decreased expression of PACS-2 reduces the integrity of MAMs and inhibits lipidation of LC3II.	[106]
